This article has been retracted.

# The influence of machine learning-based knowledge management model on enterprise organizational capability innovation and industrial development

**DOI:** 10.1371/journal.pone.0242253

**Published:** 2020-12-01

**Authors:** Zhigang Zhou, Yanyan Liu, Hao Yu, Lihua Ren

**Affiliations:** 1 Shandong University of Science and Technology, Qingdao, Shandong, China; 2 Linyi City Lanshan Economic and Information Technology Bureau, Linyi, Shandong, China; University College London, UNITED KINGDOM

## Abstract

The aims are to explore the construction of the knowledge management model for engineering cost consulting enterprises, and to expand the application of data mining techniques and machine learning methods in constructing knowledge management model. Through a questionnaire survey, the construction of the knowledge management model of construction-related enterprises and engineering cost consulting enterprises is discussed. First, through the analysis and discussion of ontology-based data mining (OBDM) algorithm and association analysis (Apriori) algorithm, a data mining algorithm (ML-AR algorithm) on account of ontology-based multilayer association and machine learning is proposed. The performance of the various algorithms is compared and analyzed. Second, based on the knowledge management level, analysis and statistics are conducted on the levels of knowledge acquisition, sharing, storage, and innovation. Finally, according to the foregoing, the knowledge management model based on engineering cost consulting enterprises is built and analyzed. The results show that the reliability coefficient of this questionnaire is above 0.8, and the average extracted value is above 0.7, verifying excellent reliability and validity. The efficiency of the ML-AR algorithm at both the number of transactions and the support level is better than the other two algorithms, which is expected to be applied to the enterprise knowledge management model. There is a positive correlation between each level of knowledge management; among them, the positive correlation between knowledge acquisition and knowledge sharing is the strongest. The enterprise knowledge management model has a positive impact on promoting organizational innovation capability and industrial development. The research work provides a direction for the development of enterprise knowledge management and the improvement of innovation ability.

## 1. Introduction

Of late years, with the development of new computer technology and big data technology, Chinese enterprises are also in rapid development; however, at the same time, the rapid development of the social economy and the intensification of market competitiveness have also brought many challenges [1, 2]. Under such an environment, if enterprises wish to continue to develop, they must adapt to the changing market environment. At present, although knowledge management has been recognized by some enterprises, the promotion and expansion of the knowledge management model needs to be improved and strengthened further [3, 4]. Taking construction enterprises as an example, most enterprises in this field have paid attention to and invested in the application of informationization construction and relevant management software. However, since most of the knowledge is stored in the human brain, regardless of the generation or flow of knowledge, it is inseparable from people’s actions, which makes the explicit transfer of knowledge in enterprises difficult to achieve. Under this background, introducing the knowledge management model into informationization construction can allow enterprises to manage knowledge more efficiently, and is expected to solve the dilemma of enterprises in knowledge management. Engineering cost management is critical to civil engineering construction, and those engineering cost consulting enterprises are responsible for engineering cost consulting management and other services. After being entrusted with relevant businesses, these enterprises can provide knowledge of economic management, laws and regulations, and intellectual services for the operation of construction and other projects. The engineering cost consulting enterprises are taken as the research object. The knowledge management model is introduced to optimize the management model of cost consulting enterprises.

Currently, it is in an information age. The rise and development of computers and network communications are changing people’s activities, such as production and life. At the same time, they are accompanied by massive amounts of data and information. Hence, the importance of data mining and analysis becomes more prominent. At present, data mining methods have been applied in sales forecasting, industry data forecasting, and chemical and medical fields. Data mining technology shows excellent performance in many fields, including knowledge maintenance and update, interactive discovery, knowledge expression and interpretation [5]. In recent years, the development of machine learning has also brought opportunities for the development of enterprises. The use of machine learning can promote the solution of many problems, and the Apriori algorithm is one of the typical representatives [6]. On this basis, data mining methods and machine learning algorithms are introduced and applied to optimize enterprise knowledge management models.

Therefore, to study the construction of the enterprise knowledge management model and promote the application of the knowledge management model in the organizational innovation capability and industrial development of the enterprises, different from previous explorations, the construction-related enterprises and engineering cost consulting enterprises are taken as examples. Through the combination of data mining techniques and machine learning methods, the correlation between various levels of knowledge management is analyzed, aiming to provide a direction for the development and application of enterprise knowledge management.

## 2. Literature review

### 2.1 Overview of knowledge management in construction enterprises and engineering cost consulting enterprises

The knowledge management model has been intensively explored by scholars. Through descriptive surveys, Khajouei and Khajouei (2017) refined the knowledge management model for identification, creation, storage, sharing, and application, and researched the knowledge management model applicable to hospitals [7]. Koohang et al. (2017) established a research model through the influence of leadership in trust, knowledge management, and organizational performance [8]. Zhang (2017) proposed a specific graph database application, which simplified the process of knowledge management, providing guidance for relevant practitioners to seek alternative methods of traditional knowledge management methods [9]. Ward et al. (2019) discussed the decision-making integration of data model of water resources system by adopting Delphi survey method, which provided a strategic view for knowledge management [10]. Yang et al. (2018) verified the model used to evaluate the relationship between task-level knowledge management and project success through structural equation modeling; it was found that when projects with unrealistic schedules experienced high levels of knowledge management, compared to more realistic projects, they were more likely to succeed [11]. Suh et al. (2017) believed that a knowledge management model that supported advanced metering networks could estimate energy consumption in the power grid environment based on the characteristics of residential buildings; this knowledge management model could be effectively applied to the management of energy demand response process of market prices and residential energy shortages [12]. Lopes et al. (2016) considered that open innovation played a key role in effective strategic sustainable management; enterprises could use knowledge management to promote sustainable innovation, which in turn, affected the sustainability of the organization [13]. In the construction industry, Lytra et al. (2020) analyzed and discussed the relationship between quality attributes and architecture design decisions of the software by reviewing and summarizing previous research results; besides, the impact of construction knowledge management methods and tools on system quality decision-making is analyzed, and the relationship between software components, uncertain factors in decision-making, and architectural knowledge management activities is revealed [14]. Antwi-Afari et al. (2018) conducted a comprehensive review and explanatory research on the critical success factors in the implementation of building information modeling, which provided a basis for the enhancement of enterprise information construction and knowledge management level [15]. Zhong et al. (2019) reviewed the research on ontology in recent years; among them, the scientometric analysis objectively reflected the current status of ontology research in the construction industry; ontology promoted the knowledge management and information retrieval of construction enterprises, and information technology enabled “knowledge management” to evolve into “building information modeling” and other models [16]. In the field of engineering cost, Meira et al. (2018) revealed the importance of a knowledge management plan in engineering cost [17].

### 2.2 Overview of management-based data mining and machine learning

For the application of data mining methods and machine learning in management models, experts and scholars have conducted corresponding researches. Lin et al. (2018) used data mining methods and machine learning technologies to study the governance model for biomass accuracy of image remote sensing algae; they revealed the excellent characteristics of fusing the two methods [18]. Gao et al. (2017) proposed a new machine learning method and applied it to the analysis and management of multimedia data [19]. Dorgo and Abonyi (2019) studied the learning event sequence of associated events in the database by introducing machine learning algorithms, which provided a direction for the management of industrial system alarms and event logs [20]. Poh et al. (2018) combined machine learning methods and data mining methods to propose a machine learning method for classifying sites based on the safety risks of construction projects; the prediction and severity assessment of accidents proved the effectiveness of the proposed method [21].

Based on the forgoing, it is found that knowledge management has applicability in many fields and can play an important role in the development and innovation of enterprises. However, there are few research works on applying data mining technology and machine learning ideas to it. At the same time, applications of the two in the fields of construction and engineering cost are rare.

## 3. Method

### 3.1 Knowledge management

The concept of knowledge management was first proposed in the 1980s, and the earliest application of this concept was among enterprises [22]. Different scholars have different views on knowledge management research, but on the whole, they are similar. In knowledge management, knowledge and management are equally important. In terms of content composition, knowledge contains tacit and explicit knowledge. Whether it is at the level of knowledge or management, the goal is to serve the enterprises. In terms of functional applications, knowledge management level plays an important role in obtaining benefits for enterprises. The realization of the entire knowledge management process is actually the integration of information, including the generation, storage, and application of knowledge. In a deeper sense, knowledge management mainly covers two levels of content, one is for information management, and the other is for human resource management; knowledge management has its uniqueness, among which the knowledge integration, intelligent development, economic resources, organizational culture, and shared innovation are the major features [23]. From the application principle, the main purpose of knowledge management is to acquire, store, and apply relevant information [24].

The realization of knowledge management is a dynamic and systematic process. From the perspective of an enterprise, knowledge management can be applied to all aspects of its management. The realization of organizational capabilities and related innovation achievements of small and medium-sized enterprises rely more on imitation learning rather than independent innovation. However, the knowledge management model is applicable to the innovation of enterprise organizational capabilities and industrial development [25]. Among them, the knowledge flow model of enterprises is shown in Fig 1 below.

**Fig 1:** Enterprise knowledge flow model.

### 3.2 Data mining based on multilayer association and machine learning

From the perspective of data mining, association rules are a key research level. Its goal is to find the minimum support threshold, minimum confidence, and effective user association rules associated with users in the object database [26, 27]. The hierarchical composition of ontology is expressed by a concept tree, in which the number of root nodes is represented by “0”; higher layers correspond to lower layers, and vice versa. For the multilayer association mining method, according to the actual situation, it can be divided into two major types. One is to use the same support level in all component layers, that is, to use a consistent minimum support threshold in each component layer, which simplifies the data collection process, but the setting of thresholds in this type is a challenging task; another is the use of successively lower levels of support in the lower levels; in this type, a variety of data collection methods can be used, such as layer-by-layer independent methods and single-item filtering methods; such setting makes this type more sensitive in the mining of multilayer data, and can reduce the generation of invalid associations [28, 29].

In data mining, ontology-based data mining (OBDM) algorithm and association analysis (Apriori) algorithm are two widely used algorithms. Among them, the OBDM algorithm can achieve high-level data mining, thereby generating high-level rules. It is formed by three sub-algorithms; the first component sub-algorithm completes normalization and generalization processing of the data granularity by using the ontology; the second component sub-algorithm is the core algorithm, including association rules and clustering algorithms; the third component sub-algorithm is a generalized combination processing for rules. In general, the OBDM algorithm uses the ontology as the springboard, which can increase the speed of data mining, and at the same time, improve the quality and effect of knowledge. In the Apriori algorithm, data mining is divided into two sub-problems; one is to find all frequent sets that meet the minimum support, and the other is to utilize the frequent sets to find all association rules that meet the minimum confidence. This kind of algorithm tool has the characteristics of fast and efficient in data mining, but it will generate many redundant rules, and its application efficiency needs to be improved further [30].

The above analysis suggests that the OBDM algorithm and the Apriori algorithm are applicable to the association rules about data mining, which can achieve high-level data mining and effective generalization of the hierarchy. However, at the same time, when these two algorithm tools are used for data mining, they are often limited to a single conceptual layer, and only a single minimum support is adopted, which brings limitations to their applications. Therefore, they are improved and optimized to propose an ontology-based multilayer association data mining algorithm, which is denoted as ML-AR algorithm. The ontology structure of data mining is Fig 2 below.

**Fig 2:** Ontology structure of data mining.

Among the improved algorithms, through the method of reducing transactions, the scanning of data volume is reduced. Assuming that there is an item set:

$$X=\left\{x_{1},x_{2},\cdots ,x_{i}\right\}$$ (1)

$$Y=\left\{y_{1},y_{2},\cdots ,y_{j}\right\}$$ (2)

Where *y*_*j*_ corresponds to the adjacent level of *x*_*i*_. Furthermore, the minimum support degree of the item set *X* is expressed by min sup(∙), and the corresponding calculation is:

$$\frac{\sum \left(S\left(y_{i}\right)/B\left(y_{i}\right)\right)}{2*R*N}+\frac{\min\;\sup\left(p+1\right)*\sum S\left(y_{i}\right)}{2*\sum \left(S\left(y_{i}\right)/B\left(y_{i}\right)\right)}$$ (3)

In (3), *S*(*y*_*i*_) represents the number of items that are not less than the minimum support threshold, *B*(*y*_*i*_) represents the number of branches, *R* represents the number of records in the database, *N* represents the number of nodes corresponding to the parent item, and *p* represents the number of layers.

On this basis, the condition that the parent item *Y* can achieve the recycling needs is:

$$\frac{S\left(y_{i}\right)}{B\left(y_{i}\right)}\geq \min\;\sup\left(p+1\right)$$ (4)

For the construction of ontology, the implementation process mainly includes the determination of the scope of the domain, the reuse of the existing ontology, the listing of the key, the definition of the class and attribute, and the definition of the attribute limitation. Taking computers and external devices as examples, the construction process of the ontology concept tree is shown in Fig 3 below.

**Fig 3:** Construction process of ontology concept tree.

To analyze and evaluate the performance of the ML-AR algorithm, Java is adopted as a development tool, and data in the University of California Irvine (UCI) dataset are chosen as experimental data to compare and analyze the proposed algorithm with the OBDM algorithm and the Apriori algorithm.

### 3.3 The construction idea of enterprise knowledge management model

For the knowledge management of enterprises, the massive data composition makes the information mismatch and low knowledge relevance during retrieval. However, in terms of the above-mentioned ontology-based association rule data mining method, due to its rich semantic composition, hierarchical relationship, and machine learning concepts, it can play an important role in the mining of knowledge data and the improvement of information matching. On this basis, considering the relative complexity of enterprise knowledge management, in the construction of the enterprise knowledge management model, the ideas of the proposed ML-AR algorithm are incorporated into it. The specific construction ideas are shown in Fig 4 below. For the construction of enterprise knowledge management model, the various components involved in knowledge management are considered, and the multilayer association rules are utilized.

**Fig 4:** The idea of constructing an enterprise management model.

### 3.4 Research design and model construction

#### (1) Questionnaire design

To clarify the actual needs of enterprises in knowledge management, the enterprises are surveyed through questionnaire. (a) The questionnaire is roughly composed of three major parts; specifically, they are the basic situation of the person being surveyed, the basic situation of the employed company, and the knowledge management of this person’s employed company. The third part is the core of the questionnaire, which can be divided into: the understanding degree of knowledge management, the knowledge acquisition, sharing, storage, and innovation, and the organization management and industry development. (b) In the part of knowledge management, according to the level of understanding, it is divided into four levels from “completely not understood” to “completely understood”, and statistical analysis of the degree of understanding of the survey participants is carried out through a percentage method. Data statistics at this level can provide a basic reference for the development direction of the enterprise knowledge management model. (c) For the level of tacit knowledge of the enterprises, the questionnaire mainly includes the proportion of senior titles of the enterprise and the proportion of the composition of the academic level. These people in the enterprise are inseparable from the level of tacit knowledge of the enterprise. (d) According to the knowledge source of the enterprises, this questionnaire starts from the two levels of work needs and other similar projects. The main topics set up include knowledge acquisition, knowledge sharing, knowledge storage, and knowledge innovation. The level of knowledge management is also the key to this questionnaire survey. (e) With regard to several levels of knowledge management, option settings include “never”, “rarely”, “frequently”, and “always”. In the knowledge management module of the questionnaire, a sample question of knowledge acquisition is “most employees of enterprises improve their professional skills and business capabilities through self-study”; a sample question of knowledge sharing is “related benefits provided by enterprises to employees”; a sample question of knowledge storage is “Enterprises build knowledge bases and train relevant personnel to promote the implementation of knowledge management”; a sample question of knowledge innovation is “Name the innovative projects developed by enterprises”. (f) This questionnaire survey is conducted through a professional website. The completed questionnaire will be sent to relevant personnel in the form of a link, which ensures the authenticity of the survey data to some extent.

#### (2) Methods and materials

This study was reviewed and approved by Natural Science Foundation of Shandong Province NO:20190615. Before the questionnaire survey, the primary content has been explained to the enterprise employees with full capacity for civil conduct. They can choose answer the question or quit this survey. The consent was informed in written and verbal.

The process of this questionnaire survey lasted from October 2019 to December 2019. A total of 125 questionnaires were finally recovered. The persons surveyed were mainly practitioners from the construction field. Among the questionnaires recovered, 50 copies were from engineering cost consulting enterprises. The entire process of questionnaire design, distribution, and data collection did not involve personal privacy. The entire questionnaire survey process was conducted with the consent of the participants; the questionnaire was not open to the public and only for research purposes. In order to test the reliability of the questionnaire, the Cronbach’s α coefficient is adopted for evaluation [31], and the validity of the questionnaire is analyzed by principal component analysis (PCA) [32].

#### (3) Construction of enterprise knowledge management model

The construction-related enterprises and engineering cost consulting enterprises are taken as research samples. Based on the results of the questionnaire survey, the construction of enterprise knowledge management models mainly includes the preprocessing of relevant data and the analysis of data correlation.

## 4. Results

### 4.1 Reliability and validity analysis results of the questionnaire

The results of the reliability and validity analysis of the questionnaire are shown in Table 1 below.

**Table 1:** Reliability and validity of the questionnaire.

Reliability	Cronbach’s α		0.848
Validity	Common factor variance	Knowledge acquisition	0.884
		Knowledge sharing	0.940
		Knowledge storage	0.718
		Knowledge innovation	0.915

The above data show that the value of Cronbach’s α in this questionnaire is above 0.8, showing that this questionnaire has excellent reliability. The extracted values of common factor variances are all higher, and the information loss is less, indicating that the overall effect of the questionnaire survey is good.

### 4.2 Performance of data mining algorithms based on multilayer association and machine learning

The comparison results of ML-AR algorithm, OBDM algorithm, and Apriori algorithm on the degree of support and the number of transactions are shown in Fig 5 below.

**Fig 5:** Comparison results of several algorithms on the number of transactions and support (In the figure, the suffix -T indicates the number of transactions, and the indicator is represented by a solid line; the suffix -S indicates the support, and the indicator is represented by a dotted line).

After analyzing the data changes, it is found that whether it is based on the number of transactions or the angle of support, the efficiency of the proposed ML-AR algorithm is superior to the OBDM algorithm and the Apriori algorithm. Specifically, under the premise that the number of transactions is small, the efficiency of several data mining algorithms is not very obvious. As the number of transactions continues to increase, the efficiency of the proposed ML-AR algorithm is significantly higher than that of the OBDM algorithm and Apriori algorithm. Finally, it shows the optimal execution efficiency; from the perspective of support, under the premise of low support, the efficiency of these data mining algorithms is also not very obvious; however, with the gradual increase in support, the efficiency of the proposed ML-AR algorithm is significantly higher than that of the OBDM algorithm and the Apriori algorithm. In the case of a higher support value, although the efficiency of the proposed algorithm has decreased, it is still superior to the OBDM algorithm and the Apriori algorithm.

### 4.3 Data processing results of the recovered questionnaires

Based on the enterprise knowledge management level, the statistical results of knowledge acquisition, knowledge sharing, knowledge storage, and knowledge innovation are shown in Fig 6 below.

**Fig 6:** Statistical results of knowledge management level.

It is shown in Fig 6 that the capabilities at all levels of knowledge management are high. In general, the proportion of knowledge storage capabilities at a weak level is 41.52%; compared to other levels, the statistical results at this level are the most unsatisfactory. Therefore, the subsequent construction of the knowledge management model will focus on this level.

Based on the four levels of knowledge management, the correlation analysis results of construction enterprises and engineering cost consulting enterprises are shown in Fig 7(A) and 7(B) below.

**Fig 7:** Correlation analysis of enterprise knowledge management level: (a) construction-related enterprises; (b) engineering cost consulting enterprises (In the figure, KA, KSh, KSt, KI represent knowledge acquisition, knowledge sharing, knowledge storage, and knowledge innovation).

After analyzing the data changes, it is found that whether for the 125 construction-related enterprises or 50 engineering cost consulting enterprises, there is a positive correlation between all levels of knowledge management; besides, from the perspective of the significance level, there is a significant positive correlation between all levels of knowledge management. Specifically, the positive correlation between knowledge acquisition and knowledge sharing is the strongest; the positive correlation between knowledge innovation and knowledge acquisition is also strong, but the positive correlation between knowledge innovation and knowledge sharing is weak.

### 4.4 Results of knowledge management model construction based on knowledge management level analysis

Combining the above analysis of data mining algorithms based on association rules and machine learning, as well as statistical analysis of knowledge management level, the knowledge management model of engineering cost consulting enterprises is initially constructed, and its schematic diagram is shown in Fig 8 below.

**Fig 8:** Knowledge management model of engineering cost consulting enterprises.

In this knowledge management model, the focus is on the organizational capacity innovation links of enterprises, as well as aspects such as knowledge application, capital investment, and related industry development. The management of knowledge is not limited to the above-mentioned levels and the engineering cost consulting industry; instead, it is also applicable in other business areas.

## 5. Discussion

The reasons to the above results are that when the value of the support is at a low level, the support in the current situation is greater than the support of the parent, the selection of support at this time does not match the actual data. This also shows from the side that the algorithm needs to be considered in the selection of support further. If the value of support is too high or too low, the performance of the algorithm will be affected. The proposed data mining algorithm incorporates association rules and machine learning into the knowledge, and is expected to be applied to the enterprise knowledge management model, which can promote the development of enterprise knowledge management capabilities. Knowledge management involves massive amounts of data. Ontology-based multilayer association rules and machine learning data mining methods are of great significance in the development of enterprise knowledge management models.

The above analysis reveals that if the sharing level of knowledge management needs enhancing, it is necessary to first increase the level of access to knowledge management. Although the positive correlation between the innovation level and the sharing level of knowledge management is not strong, it is obvious that the enterprise knowledge management model is also of great significance for organizational capability innovation and industrial development, including knowledge sharing and knowledge acquisition, which cannot be ignored. This is consistent with the results of Cillo et al. (2019), who took agricultural product enterprises as examples and explored the relationship between knowledge management capabilities and successful open innovation [33]. Although some differences are found in production and operation models between agricultural product enterprises and the construction enterprises and engineering cost consulting enterprises, the profound relationship between knowledge management capabilities and innovation is potentially consistent. Based on previous results, the ideas of data mining and machine learning are incorporated, which is an important innovation that is different from previous works. In general, enterprises must realize the innovation of organizational capabilities through the knowledge management model and promote the development of related industries; therefore, it is crucial for the integration and coordination of all levels of knowledge management. For example, in the knowledge acquisition stage, it is necessary to be proficient in engineering construction projects such as project type and structure scale. Meanwhile, the necessary data are recorded, and the basic situation of project participants is mastered. Although the task integration and perfection of this link cannot totally guarantee the complete completion of the project, it can also make related projects achieve double the effect with half the effort. Similarly, for all other levels, it is also necessary to improve integration so that the integration and coordination can enable and improve the organization’s organizational innovation capabilities and industrial development [34].

## 6. Conclusion

The construction-related enterprises and engineering cost consulting enterprises are taken as the research samples, the data mining algorithm ML-AR is introduced, the collected data are analyzed and characterized in the form of questionnaires, and the knowledge management model for engineering cost consulting enterprises is built. The results show that the reliability and validity of this questionnaire survey are excellent. Also, the proposed ML-AR algorithm has high efficiency; especially, when the number of transactions and support are at a high level, the efficiency of the ML-AR algorithm is more significant. There is a significant correlation between all levels of knowledge management. Among them, the positive correlation between knowledge acquisition and knowledge sharing is the strongest, followed by knowledge innovation, while the correlation between knowledge innovation and knowledge sharing is weak. This provides a possible idea for the construction of the enterprise knowledge management model, which is expected to be applied in promoting organizational innovation capabilities and industrial development.

However, the research on the enterprise knowledge management model is still in the exploration stage, and the selection of research samples is not comprehensive enough. The knowledge management model only provides a general direction for the organization of enterprises and the development of the industry; At the same time, the knowledge storage capacity at a weak level has not been detailed and analyzed further. In the future, the research sample will be expanded, and the research on knowledge management models in organizational capability innovation and industrial development will be deepened.

## Supporting information

S1 Data (RAR)
